This article has been retracted.

# ING5‐mediated antineuroblastoma effects of suberoylanilide hydroxamic acid

**DOI:** 10.1002/cam4.1634

**Published:** 2018-08-09

**Authors:** Ji‐cheng Wu, Hua‐mao Jiang, Xiang‐hong Yang, Hua‐chuan Zheng

**Affiliations:** ^1^ Tumor Basic and Translational Laboratory The First Affiliated Hospital of Jinzhou Medical University Jinzhou China; ^2^ Department of Pathology Shengjing Hospital of China Medical University Shenyang China

**Keywords:** histone acetylation, ING5, miRNA, neuroblastoma, suberoylanilide hydroxamic acid

## Abstract

Neuroblastoma is the most common extracranial solid neuroendocrine cancer and is one of the leading causes of death in children. To improve clinical outcomes and prognosis, discovering new promising drugs and targeted medicine is essential. We found that applying Suberoylanilide hydroxamic acid (SAHA; Vorinostat, a histone deacetylase inhibitor) and MG132 (a proteasome inhibitor) to SH‐SY5Y cells synergistically suppressed proliferation, glucose metabolism, migration, and invasion and induced apoptosis and cell cycle arrest. These effects occurred both concentration and time dependently and were associated with the effects observed with inhibitor of growth 5 (ING5) overexpression. SAHA and MG132 treatment increased the expression levels of ING5, PTEN, p53, Caspase‐3, Bax, p21, and p27 but decreased the expression levels of 14‐3‐3, MMP‐2, MMP‐9, ADFP, Nanog, c‐myc, CyclinD1, CyclinB1, and Cdc25c concentration dependently, similar to ING5. SAHA may downregulate miR‐543 and miR‐196‐b expression to enhance the translation of ING5 protein, which promotes acetylation of histones H3 and H4. All three proteins (ING5 and acetylated histones H3 and H4) were recruited to the promoters of *c‐myc, Nanog, CyclinD1, p21,* and *p27* for complex formation, thereby regulating the mRNA expression of downstream genes. ING5 overexpression and SAHA and/or MG132 administration inhibited tumor growth in SH‐SY5Y cells by suppressing proliferation and inducing apoptosis. The expression of acetylated histones H3 and ING5 may be closely linked to the tumor size of neuroblastomas. In summary, SAHA and/or MG132 can synergistically suppress the malignant phenotypes of neuroblastoma cells through the miRNA‐ING5‐histone acetylation axis and via proteasomal degradation, respectively. Therefore, the two drugs may serve as potential treatments for neuroblastoma.

## 1 INTRODUCTION

Neuroblastoma is the most common extracranial solid neuroendocrine cancer, accounting for 6%‐10% of all childhood cancers and 15% of cancer deaths in children. This cancer can arise from any neural crest element of the sympathetic nervous system in childhood, with nearly half of cases occurring in children under the age of 2. It most often originates in one of the adrenal glands, but it can also develop from nerve tissues in the neck, chest, abdomen, or pelvis.^1^, ^2^ Therefore, to improve clinical outcomes and prognosis, discovering new promising drugs and targeted agents is essential.

Histone deacetylases (HDACs) and histone acetyltransferases (HATs) work together as transcriptional corepressors and activators to regulate gene expression by transforming nucleosome conformation and changing the stability of several large transcription factor complexes.^3^, ^4^ Suberoylanilide hydroxamic acid (SAHA) is a synthetic hydroxamic acid with a zinc atom at the bottom of its catalytic cavity. SAHA arrests cancer cell growth by inhibiting classes I and II zinc‐binding HDACs.^5^, ^6^ Substantial evidence indicated that SAHA induced histone acetylation in transcription factor complexes that regulate the genetic expression of molecules associated with malignant phenotypes.^7^ Similar to HDACi, ING5 may form MOZ/MORF‐BRPF1/2/3‐ING5‐hEaf6 and JADE1/2/3‐HBO1‐ING4/5‐hEaf6 HAT complexes to acetylate histones H3 and H4, respectively.^8^

Suberoylanilide hydroxamic acid suppresses the growth of HeLa cells and induces apoptosis, which is accompanied by PARP cleavage, Caspase‐3 activation, potential loss of the mitochondrial membrane, and ROS generation.^9^ It also suppresses the growth of paclitaxel‐resistant ovarian cancer cells by decreasing the expression of the endogenous genes *Bcl‐2* and *c‐myc* and increasing the expression of *Bax*.^10^ Ding et al^11^ found that SAHA triggered the mesenchymal‐epithelial transition but induced Akt phosphorylation of PC3 and A549 cells in an HGF‐independent manner, which is partially involved in the resistance of solid tumors to SAHA. In addition, SAHA epigenetically regulates the miR‐17‐92 cluster and MCM7 to enhance the expression of MICA in hepatoma cells.^12^ In CAL27 and SCC25 cells, SAHA treatment significantly increases the expression of tumor suppressors miR‐107 and miR‐138 but decreases the expression of oncogenes PKCε, HIF1β, CDK6, and RhoC.^13^ Wolf et al^14^ demonstrated that SAHA specifically inhibited the expression of xCT‐transporter to produce tumor cell stress, allowing xCT equilibration and leading to a normalized tumor microenvironment.

In neuroblastoma cells, SAHA decreased cell viability through apoptotic induction.^15^ A quantitative proteomics study demonstrated that SAHA treatment in SH‐SY5Y cells led to altered protein expression of histone lysine acetylation and butyrylation.^16^ In this study, we explored the effects of SAHA on biological phenotypes (eg, proliferation, apoptosis, cell cycle, glucose metabolism, migration, and invasion) and its synergistic effects with MG132 (a proteasome inhibitor) and subsequently screened the phenotype‐related molecules of neuroblastoma cells in vivo and in vitro. In addition, we analyzed the underlying molecular mechanisms involved in these effects.

## 2 MATERIALS AND METHODS

### 2.1 Cell lines and transfection

Neuroblastoma cells (SH‐SY5Y, SK‐N‐AS, NGP, and SK‐N‐BE2) were kindly gifted by Professor Carol J Thiele from the National Institutes of Health, National Cancer Institute, USA, and cultured in Dulbecco's modified Eagle's medium (GIBCO, Shenyang, China) supplemented with 10% fetal bovine serum (GIBCO). The cells were incubated in 5% CO_2_ humidified atmosphere at 37°C. The plasmid pEGFP‐N1‐ING5, pEGFP‐N1 vector (mock), and miR mimics and inhibitors (Table S1) were transfected in the cells 24 hours after seeding on dishes. All cells were collected by centrifugation, washed twice with phosphate‐buffered saline (PBS), and used for the subsequent experiments.

### 2.2 Cell proliferation

Cell Counting Kit‐8 (CCK‐8; Dojindo, Kumamoto, Japan) was applied to define the number of viable cells in 96‐well plates by measuring the absorbance at 450 nm. Additionally, cells were seeded in specially designed 16‐well E‐plates, and the xCELLigence assay was used to continuously monitor cell viability with the xCELLigence System (ACEA Biosciences, Hangzhou, China).

### 2.3 Cellular energy metabolism

The cellular energy metabolism assay (Seahorse Bioscience, USA) was used to measure mitochondrial respiration and glycolysis. The rates of oxygen consumption (OCR) and extracellular acidification (ECAR) were measured as the rates of respiration and glycolysis, respectively. Briefly, 2.0 × 10^4^ cells were seeded in 24‐well plates, and several agents were added in the following order: 10 mmol/L glucose, 1.5 μmol/L oligomycin (to block ATP synthase to assess respiration requirements for ATP turnover), and 50 mmol/L 2‐DG for the glycolysis assay, and 1.5 μmol/L oligomycin, 2 μmol/L FCCP (a proton ionophore that induces chemical uncoupling and maximal respiration), 0.5 μmol/L Rotenone and antimycin A (to completely inhibit electron transport to measure nonmitochondrial respiration) were injected for the mitochondrial respiration assay. The OCR and ECAR values were measured from 3 wells per sample, and the experiments were repeated three times.

### 2.4 Cell cycle analysis

The cells were harvested by trypsinization, rinsed twice with PBS, and fixed in 5 mL of 70% ice‐cold ethanol for more than 2 hours. Then, the cells were resuspended in 1 mL of PBS containing 200 mg/mL RNase at 37°C for 1 hour. The cells in the tube were pelleted, resuspended in propidium iodide (PI) at a concentration of 50 μg/mL, and incubated in the dark at room temperature for 30 minutes. Cell cycle analysis was performed by PI staining and flow cytometry. Modfit software was used to analyze changes in the cell cycle.

### 2.5 Apoptosis assay

Flow cytometry was executed by staining with PI and FITC‐labeled Annexin V (KeyGEN Biotech, Beijing, China) following the manufacturer's instructions. Briefly, cells were harvested by trypsinization (without ethylenediaminetetraacetic acid), rinsed twice with PBS and stained with FITC‐labeled Annexin V at room temperature for 30 minutes. Apoptotic cells were measured by phosphatidylserine staining externalization (Annexin V binds to phosphatidylserine). Then, the cells were stained with propidium iodide (PI) at a concentration of 50 μg/mL and incubated in the dark at room temperature for 30 minutes. The cell apoptosis assay was examined by flow cytometry. FlowJo software was used to analyze changes in apoptosis.

### 2.6 Wound healing and transwell assays

Cells were seeded in 6‐well culture plates at a density of 1.0 × 10^6^. After reaching confluence, the cell monolayer in each well was scratched with a pipette tip, washed three times with PBS, and cultured in FBS‐free medium. Cells were photographed after 24 hours, and the scratch area was measured using ImageJ software. For the invasion assay, 1 × 10^5^ cells were resuspended in serum‐free DMEM and seeded into the upper chamber of Matrigel‐coated transwell inserts (BD Bioscience, USA). The lower compartment of the chamber contained 10% FBS as a chemoattractant. After incubation for 24 hours at 37°C in the incubator supplemented with 5% CO_2_, the noninvasive cells on the upper surface of the chamber were wiped away with a cotton swab, and the cells adhered to the lower membrane were fixed with 4% formaldehyde in PBS and stained with crystal violet to quantify the extent of invasion.

### 2.7 Chromatin immunoprecipitation (ChIP)

ChIP assays were performed with a ChIP assay kit (MILLIPORE Magna ChIPTM G) according to the manufacturer's instructions. Briefly, cells were cross‐linked with 1% formaldehyde and collected in lysis buffer. Chromatin was then digested with Micrococcal Nuclease. Immunoprecipitation was incubated with 3 μg of acetyl‐histone H3, acetyl‐histone H4, and ING5 antibody or normal mouse IgG followed by immunoprecipitation with Protein G Agarose Beads during an overnight incubation at 4°C with gentle shaking. As an input reference, 2% were removed before antibody supplemental and stored at ‐20°C. The ChIP DNA was reverse‐cross‐linked with 5 mol/L NaCl and Proteinase K and then purified. Immunoprecipitated DNA was amplified by PCR using primers. The primers of each PCR set, the sizes of PCR products, and annealing temperatures have been described previously.^17^ Coimmunoprecipitation of double ChIP was performed using acetyl‐histone H3, and then, ING5 or acetyl‐histone H4 in ING5 transfectants.

### 2.8 Coimmunoprecipitation (Co‐IP)

Cell lysates containing at least 1000 μg of protein from each sample were precleared with 50 μL of protein A‐Sepharose beads for 1 hour at 4°C and incubated with 5 μg of ING5, Ac‐H3, or Ac‐H4 antibody in a 1‐mL mixture overnight at 4°C on a rotator. Then, 100 μL of protein A‐Sepharose beads (50% slurry) were added and rotated at 4°C for 3 hours. The beads were then centrifuged and washed 5 times with 1% NP40 lysis buffer. The precipitates were eluted by adding 50 μL of 1 × sample loading buffer and boiled. The supernatant obtained after centrifugation was subjected to Western blot analysis.

### 2.9 Selection of patient samples

Pathological blocks of neuroblastomas were collected from patients undergoing complete surgical resection as an initial treatment between January 2003 and December 2013 at Shengjing Hospital of China Medical University (n = 50). The average age of the patients at the time of surgery was 6.6 years (range 0.6‐21 years), and median tumor size was 63 mm. None of the patients had undergone chemotherapy or radiotherapy prior to surgery. Written informed consent was provided by the patients’ guardians, and the study was approved by Clinical Research Ethics Committee of the First Affiliated Hospital of Jinzhou Medical University.

### 2.10 MicroRNA prediction and transfection

We used the bioinformatics databases TargetScan and miRanda to predict the microRNAs that could potentially combine with *ING5* mRNA, and then, we commissioned a company (GenePharma, Shanghai, People's Republic of China) to synthesize the mimics and inhibitors. Cells were seeded into 6‐well plates until they reached 50%‐70% confluence and were then transfected with microRNAs using Lipofectamine 3000 reagent (Life Technologies Corporation, Carlsbad, CA) according to the manufacturer's instructions.

### 2.11 Pathology and tissue microarray (TMA) analysis

All tissues used in this study were subjected to routine block preparation, cut into thin slides, and stained with hematoxylin and eosin (H&E) for histological analysis. The clinicopathological and pathological staging values were evaluated for neuroblastoma samples according to the TNM staging system and the World Health Organization (WHO) classification system. TMA was prepared using a Tissue Microarrayer (AZUMAYA KIN‐1, Tokyo, Japan).

### 2.12 Xenograft model

BALB/c nude mice (male, 4‐6 weeks) were purchased from the Beijing Huafukang Bioscience Co. Inc. (Beijing) and kept in a specific pathogen‐free (SPF) facility with a 12‐h light/dark cycle. All experimental procedures were approved by the Animal Experiment Ethical Statement of Jinzhou Medical University. SH‐SY5Y cells or their ING5 transfectants were injected into the axilla of the mice. When the tumor diameter reached 8 mm, 20 mg/kg SAHA, 2 mg/kg MG132, or 10 mg/kg SAHA + 1 mg/kg MG132 was intraperitoneally injected into the mice from the 9th, 12th, and 15th days of cell injection. Tumor growth was then monitored for 18 days and calculated using the equation (Length*Wide^2^)/2. At the end of the experiment, mice from each group were anesthetized, photographed, and sacrificed for further analysis.

### 2.13 Real‐time reverse transcriptase‐polymerase chain reaction (real‐time RT‐PCR)

Total RNA was isolated from cancer cells using TRIzol (Takara, Kyoto, Japan). Reverse transcription was performed from 2 μg of total RNA using AMV reverse transcriptase random or specific primers (Table S1). The PCR primers used in this study were designed according to the sequences in GenBank as previously described^17^ or shown in Table S2. Amplification of cDNA was performed in accordance with the SYBR Premix Ex Taq II kit (Takara). GAPDH was used as an internal control.

### 2.14 Western blot analysis

Protein assays were performed by the Bradford method using the Bio‐Rad protein assay kit (Bio‐Rad, USA). Western blot analysis was carried out as previously described.^17^ The primary antibodies are shown in Table S3.

### 2.15 Immunohistochemistry

Consecutive sections of tissue samples were deparaffinized with xylene, rehydrated with alcohol, and subjected to intermittent irradiation immunohistochemistry as previously described.^17^ Negative controls were prepared by omitting the primary antibody. The classification standard of the dyeing results was as follows: 1 = 1%‐49%; 2 = 50%‐74%; and 3 ≥ 75%. Staining intensity was defined as follows: 0 = negative; 1 = weak; 2 = moderate; and 3 = strong. Positive expression and the staining intensity of each protein were multiplied to obtain the final score: − was equal to 0 points; + was equal to 1 or 2 points; + + was equal to 3‐5 points; and + + + was equal to 6‐9 points. Three independent observers (WJC, JHM and ZHC) evaluated the results as previously reported.^17^

### 2.16 Terminal deoxynucleotide transferase‐mediated dUTP nick labeling (TUNEL)

TUNEL was performed using the Apoptosis Detection Kit (Millipore, USA) according to the manufacturer's instruction. Briefly, paraffin‐embedded sections were incubated with proteinase K at 37°C for 45 minutes. Endogenous peroxidase activity was blocked by incubation with 3% hydrogen peroxide in methanol. Paraffin sections were washed three times with PBS and then subjected to TUNEL staining. Conjugated horseradish peroxidase was visualized with DAB, followed by counterstaining with methyl green.

### 2.17 Statistical analysis

All experiments were repeated independently at least three times, and data are presented as mean ± standard deviation. Statistical tests for data analysis included the one‐way analysis of variance and Student's 2‐tailed *t* test. Bivariate correlations between study variables were calculated by Spearman's rank correlation coefficients. *P* values of .05 or less were considered statistically significant. The statistical analyses were performed using the SPSS 17.0 statistical software package.

## 3 RESULTS

### 3.1 Antitumor effects of SAHA and/or MG132 on the phenotypes of SH‐SY5Y cells

To investigate the inhibitory effects of SAHA and/or MG132 on aggressive phenotypes, we treated neuroblastoma SH‐SY5Y cells with both reagents to screen proliferation, apoptosis, glucose metabolism, invasion, and metastasis. SAHA and MG132 were found to reduce SH‐SY5Y cell proliferation both time and dose dependently according to the CCK‐8 and xCELLigence assays (Figure 1A,B, *P* < .05). In addition, SAHA and MG132 exposure apparently inhibited cell energy metabolism (Figure 1C, *P* < .01), induced G_1_ arrest (Figure 1D, *P* < .05), and promoted apoptosis (Figure 1E, *P* < .05) in a concentration‐dependent manner. Wound healing and transwell invasion assays demonstrated that SAHA and MG132 exposure decreased cell migration and invasion in a concentration‐dependent manner (Figure 1F,G, *P* < .05). In addition, SAHA and MG132 synergistically induced cell cycle arrest, promoted apoptosis, inhibited proliferation, cell migration, and invasion, and suppressed cellular energy metabolism in SH‐SY5Y cells. To clarify the molecular mechanisms, we performed Western blot to screen the phenotype‐related proteins. As shown in Figure 1H, SAHA and/or MG132 treatment upregulated the expression of ING5, PTEN, p53, Caspase‐3, Bax, p21, and p27 and downregulated the expression of 14‐3‐3, MMP‐2, MMP‐9, ADFP, Nanog, c‐myc, CyclinD1, CyclinB1, and Cdc25c. Interestingly, SAHA treatment enhanced the acetylation of histones H3 and H4; however, this effect was not observed with MG132 exposure.

**Figure 1:** Effects of SAHA and MG132 on the biological events of SH‐SY5Y cells. Cell proliferation was determined by CCK‐8 (A) and xCELLigence assays (B). The cellular energy metabolism assay detected the rate of oxygen consumption (OCR) and extracellular acidification (C). Flow cytometric analysis was used to detect the cell cycle (D) and apoptotic induction (E). Wound healing (F) and Transwell assays (G) were used to detect the migration and invasion abilities of SH‐SY5Y cells. The protein expression levels of phenotypes were screened by Western blot (H). Note: S0.2, SAHA 0.2 μmol/L; M0.3, MG132 0.3 μmol/L; S0.5, SAHA 0.5 μmol/L; M0.6, MG132 0.6 μmol/L; S0.2+ M0.3, SAHA 0.2 μmol/L and MG132 0.3 μmol/L. *P < .05 vs the treatment group. Each bar represents the mean ± standard deviation of three experiments, with the control as “1.” *P < .05 vs SAHA/MG132 treatment

### 3.2 Influence of ING5 overexpression on the phenotypes of SH‐SY5Y cells

To study the role of ING5, we successfully transfected its GFP‐tagged plasmid into SH‐SY5Y cells, as demonstrated by RT‐PCR and Western blot (Figure 2A). Compared to the control and mock conditions, ING5 overexpression decreased cell viability, SAHA chemosensitivity, and cell glucose metabolism and induced apoptosis (Figure 2B‐D, *P* < .05). PI staining indicated that ING5 overexpression resulted in G_2_ arrest of SH‐SY5Y cells (Figure 2E, *P* < .05). Based on wound healing and transwell chamber assays, cell migration and invasion were weakened in ING5 transfectants (Figure 2F,G, *P* < .05). The expression of phenotype‐related proteins was the same in ING5 transfectants as in SAHA‐treated SH‐SY5Y cells (Figure 2H).

**Figure 2:** Effects of ING5 overexpression phenotypes in SH‐SY5Y cells. After transfection of pEGFP‐N1‐*ING5*, ING5 expression became strong in SH‐SY5Y cells as indicated by RT‐PCR and Western blot (A). The transfectants showed low growth, chemoresistance to SAHA (B), low glucose metabolism (C), G_1_ arrest (D), and higher levels of apoptosis (E) compared with the control and mock conditions. Invasion and migration abilities were weaker in the ING5 transfectants than those observed under the control and mock conditions according to wound healing (F) and Transwell chamber assays (G). The protein expression levels of the phenotypes were screened by Western blot (H). Each bar represents the mean ± standard deviation of three experiments, with the control as “1.” *P < .05 vs the *ING5* transfectants

### 3.3 Effects of SAHA treatment on transcription regulation of associated genes in SH‐SY5Y cells

To explore the transcription regulation of the genes associated with phenotypes after SAHA treatment and ING5 overexpression, we examined the protein‐protein and protein‐DNA interactions of effectors (acetylated histones and ING5). As shown in Figure 3A, acetyl‐histone H3 (Ac‐histone H3), acetyl‐histone H4 (Ac‐histone H4), and ING5 were found to bind to the special fragments of *p21, p27, c‐myc, CyclinD1,* and *Nanog* promoters. Therefore, SAHA treatment and ING5 overexpression may be involved in recruiting more Ac‐histone H3, Ac‐histone H4, and ING5 proteins to these promoters. A Co‐IP assay conducted in SH‐SY5Y cells revealed that the interaction between Ac‐histone H3, Ac‐histone H4, and ING5 was strengthened by SAHA exposure and ING5 overexpression (Figure 3B). Double‐ChIP assay indicated that Ac‐H3 bound to Ac‐H4 or ING5 in the promoters of *p21, p27,* and *c‐myc* (Figure 3C). Additionally, SAHA treatment and ING5 overexpression decreased the mRNA expression of *c‐myc, Nanog,* and *CyclinD1* but increased the mRNA expression of *p27*and *p21* (Figure 3D).

**Figure 3:** Molecular mechanisms underlying SAHA/MG132 treatment effects. The promoter binding sites of ING5, acetyl‐histone H3 (Ac‐H3) and H4 (Ac‐H4) were determined by a ChIP assay targeting *p21*,* p27*,* Cyclin D1*,* c‐myc,* and *Nanog* (A). The interaction between ING5, Ac‐H3, and Ac‐H4 was examined by Co‐IP assay and Western blot (B). Double ChIP was performed by acetyl‐histone H3 and then ING5 or acetyl‐histone H4 using ING5 transfectants (C). Transcriptional control gene expression was detected by real‐time RT‐PCR (D). M: DNA marker; ND: No DNA control; NC: negative control; PC: positive control; S 0.5, SAHA treatment (0.5 μmol/L); ctr, control; C11, clone 11

### 3.4 Effects of SAHA on miRNAs and subsequent ING5 expression of SH‐SY5Y cells

To explore how SAHA increases the expression of ING5, we consulted the literature and focused on transcription regulation. As microRNA is the classical transcription factor, we conducted microRNA experiments to explore the mechanism of SAHA. Through microRNA software, we predicted that miR‐640, miR‐543, miR‐624‐3p, and miR‐196‐b target *ING5* mRNA (Figure 4A). We hypothesized that SAHA may upregulate ING5 expression through these miRNAs. Through real‐time RT‐PCR, we determined that SAHA exposure reduced the expression of these miRNAs (Figure 4B). To further demonstrate this effect, we successfully transfected mimics and inhibitors of the four miRNAs into SH‐SY5Y cells and found that SAHA exposure decreased the expression of these miRNAs in these transfectants (Figure 4C). Only miR‐543 and miR‐196‐b overexpression decreased ING5 protein expression in SH‐SY5Y cells, while SAHA may ameliorate inhibition. Opposite effects were observed for their inhibitors (Figure 4D).

**Figure 4:** Effects of SAHA exposure on ING5 expression through miRNA expression downregulation in SH‐SY5Y cells. The target sites of miRNAs for ING5 mRNA were forecasted by miRNA software (A). SAHA treatment lowered miR‐640 (640), miR‐543 (543), miR‐624‐3p (624), and miR‐196‐b (196) expression in SY5Y cells as indicated by real‐time PCR (B). We successfully transfected mimics and inhibitors of the four miRNAs into SH‐SY5Y cells and found that SAHA exposure decreased miRNA expression (C). Western blot showed that both miR‐543 and miR‐196‐b overexpression decreased ING5 protein expression in SY5Y cells, but SAHA ameliorated this inhibition. The opposite effects were observed for their inhibitors (D). Note: S, SAHA treatment; mm, mimics; in, inhibitors. Each bar represents the mean ± standard deviation of three experiments, with the control as “1”. *P < .05 vs the control; #,*P* < .05 vs no SAHA treatment

### 3.5 Effects of SAHA on the miRNA/ING5/acetyl‐histone pathway of SK‐N‐AS, NGP, and SK‐N‐BE2 cells

To confirm the miRNA/ING5/acetyl‐histone pathway in neuroblastoma cells, we selected another three cell lines (SK‐N‐AS, NGP, and SK‐N‐BE2) to investigate the molecular effects of SAHA. SAHA exposure was found to significantly inhibit viability both concentration and time dependently (Figure 5A, *P* < .05). Additionally, SAHA treatment caused downregulated expression of miR‐543 and miR‐196‐b in these cell lines (Figure 5B, *P* < .05). Overexpression of ING5, Ac‐H3, Ac‐H4, p21, and p27 and underexpression of CyclinD1, CyclinB1, c‐myc, and Nanog were observed in the three cell lines after exposure to SAHA (Figure 5C).

**Figure 5:** Effects of SAHA on the miRNA/ING5/acetyl‐histone pathway in SK‐N‐AS, NGP and SK‐N‐BE2 cells. SAHA significantly suppressed the cell viability of neuroblastoma cells concentration and time dependently (A, *P* < .05). The expression levels of miRNAs, ING5, acetyl‐histones, p21, p27, CyclinD1, c‐myc, and Nanog were screened by real‐time PCR (B) and Western blot (C). *P < .05 vs the treatment groups

### 3.6 Effects of SAHA and/or MG132 treatment and ING5 transfectants on the tumor growth of SH‐SY5Y cells

Subsequently, we evaluated the effects of SAHA and/or MG132 exposure and ING5 overexpression on tumor growth in a xenograft mouse model of neuroblastoma.. The tumor volumes of SH‐SY5Y xenografts were smaller than those of controls with SAHA or MG132 treatment alone, while a synergistic effect was observed when the treatments were combined (Figure 6A, *P* < .05). ING5 overexpression elicited the same results as SAHA treatment (Figure 6A, *P* < .05). To confirm the molecular mechanisms, we performed Western blot, immunohistochemistry, and TUNEL using xenograft tumor samples. Under both SAHA treatment and ING5 overexpression conditions, neuroblastoma cells exhibited higher expression levels of acetyl‐histones H3 and H4, p21, p27, p53, PTEN, Bax, and LC‐3B compared to the controls. The opposite effect was observed for Nanog, CyclinD1, c‐myc, CyclinB1, Bcl‐2, 14‐3‐3, MMP‐2, MMP‐9, ADFP, and Cdc25c (Figure 6B). In addition, Ki‐67 immunostaining and TUNEL assay demonstrated that the inhibitory effect had positive correlations with low proliferation and high apoptosis compared with the controls (Figure 6C).

**Figure 6:** Effects of SAHA and/or MG132 and ING5 overexpression in vivo. After SAHA and/or MG132 exposure or ING5 overexpression, SH‐SY5Y cell growth was determined by measurements of growth curves and tumor volumes and weights (A). Phenotype‐related proteins were screened by Western blot in xenograft tumors (B). Immunohistochemistry and TUNEL were employed to examine proliferation, apoptosis, and the expression levels of relevant proteins (C). Note: SAHA, 20 mg/kg; MG132, 2 mg/kg; SAHA (S) +MG132 (M), SAHA 10 mg/kg and MG132 1 mg/kg. *P < .05 vs the treatment groups

### 3.7 Associations of acetyl‐histones and ING5 expression with clinicopathological parameters of neuroblastoma

Due to the importance of acetyl‐histones and ING5 to the antitumor effects of SAHA, we detected their expression and analyzed their clinicopathological significance in neuroblastoma samples. Immunohistochemistry revealed that the acetylated histones H3 and H4 were predominantly expressed in the nuclei of neuroblastoma cells, while ING5 was found in the cytoplasm or nucleus (Figure 7A). Ac‐histone H3 or cytoplasmic ING5 expression was positively linked to neuroblastoma tumor size (*P* < .05, Figure 7B). Nuclear ING5 expression was negatively linked to neuroblastoma tumor size (*P* < .05, Figure 7B).

**Figure 7:** Expression of acetyl‐histones and ING5 in neuroblastoma. Ac‐histones H3 (Ac‐H3) and H4 (Ac‐H4) were localized to the nuclei of neuroblastoma cells, while ING5 was found in the cytoplasm and/or nucleus (A). The expression levels of acetyl‐histone H3 and ING5 were compared with neuroblastoma tumor size (B). *p < 0.05 vs Tumor size ≥ 6.3 cm.

## 4 DISCUSSION

The most successful clinical application of HDACis were the SAHA and romidepsin, which have been approved by FDA to be used for refractory cutaneous and peripheral T‐cell lymphoma.^18^ In addition to these two agents, the butyrates, valproic acid, and newer compounds such as panobinostat, givinostat, mocetinostat, belinostat, and pracinostat have been extensively studied in the clinic with varying results.^19^, ^20^, ^21^ Although some of these agents often demonstrate more potent antitumor effects than SAHA and romidepsin in preclinical testing, none have thus far demonstrated vastly superior clinical activity, or more favorable toxicity profiles, and accordingly none have yet been registered for clinical use except panobinostat (registered in FDA and EMEA). The antineoplastic effects of SAHA have been observed in various malignancies.^9^, ^10^, ^11^, ^12^, ^13^, ^14^, ^15^, ^17^, ^22^, ^23^, ^24^, ^25^, ^26^, ^27^, ^28^ In advanced leukemia and myelodysplastic syndrome, SAHA exposure induced significantly lower antileukemia activity than the maximum tolerated dose and inhibited the HDAC activity of peripheral blood and bone marrow blasts.^29^ Foster et al^30^ found that co‐administration of Bcl‐2 inhibitor ABT‐737 and SAHA induced apoptosis accompanied by Noxa upregulation, Bax activation, and mitochondrial dysfunction in PTEN‐intact glioma cells. SAHA/Parthenolide combination promoted GSH depletion, Δψm reduction, and cytochrome c release and activated Caspase‐3 via histones H3 and H4 hyperacetylation or downregulated DNMT1 expression.^25^ SAHA and 5‐FU synergistically inhibited the proliferation of hepatocellular carcinoma cells by inducing G_0_/G_1_ arrest and caspase‐dependent apoptosis.^24^ Cisplatin and SAHA dose dependently and synergistically reduced the viability of cholangiocarcinoma cells and induced cell apoptosis, accompanied by upregulation of p53 and p21 and downregulation of CDK4 and Bcl‐2.^22^

In this study, we confirmed that SAHA and MG132 inhibited cell viability, energy metabolism, migration, and invasion and induced apoptosis and G_1_ arrest in SH‐SY5Y cells. MG132 and SAHA demonstrated a synergetic effect, suggesting that their combination may enhance neuroblastoma treatment. Additionally, a novel discovery in this study is that SAHA and/or MG132 may noticeably inhibit neuroblastoma growth in tumor‐bearing mice as evidenced by proliferation inhibition and apoptotic induction. These effects were also observed in glioma^17^ and gastric^26^ cancer cells when exposed to both SAHA and MG132. Recent evidence suggested that SAHA and XL184 synergistically promoted cell apoptosis and markedly inhibited tumor growth in prostate and lung cancer cells.^11^ Consistent with our results, SAHA combined with cisplatin or decitabine can reinforce the antitumor effect on oral squamous cancer cells.^31^ MG132 combined with cisplatin or arsenic trioxide can enhance the drug sensitivity of ovarian cancer^32^ or Raji cells.^33^ Considering these findings, SAHA and MG132 can be used synergistically to eliminate neuroblastoma cells.

Reportedly, both p21 and p27 can interact with the Cyclin‐CDK complex to reduce cells in the G_1_ phase.^34^ SAHA and/or MG132 treatment decreased the expression of *CyclinD1* at the mRNA and protein levels. Conversely, p21 expression was increased in neuroblastoma cells, accounting for G_1_ arrest. The *Cdc25C* gene contains *p53* binding sites, while p53 serves as a master switch that coordinates stress signals associated with apoptosis and cell cycle arrest.^35^, ^36^ CyclinB1 can interact with Cdk1 and is subsequently involved in the early progress of mitosis.^37^ Our results revealed that the protein expression levels of CyclinB1 and Cdc25C were significantly decreased by SAHA and/or MG132 treatment, accounting for their reduction of G_2_‐phase cells. Cell apoptosis was promoted by the translocation of Bax to the mitochondria, followed by Caspase‐3 activation.^38^ The apoptotic induction capacity of SAHA and/or MG132 was observed through upregulated Bax and Caspase‐3 expression. MMP overexpression promoted cancer metastasis by breaking down the extracellular microenvironment,^39^ and Nanog is a stem cell transcription factor that is crucial for malignant transformation and progression.^40^ Our study also indicated that SAHA or/and MG132 suppressed the migration and invasion of neuroblastoma cells by decreasing the expression of MMP‐2, MMP‐9, and Nanog in SH‐SY5Y cells. PTEN acts as a specific protein‐phospholipid phosphatase to inhibit the Ras/MAPK and Akt/PKB pathways.^39^ Upregulation of both tumor suppressors was also responsible for the antitumor effects of SAHA/MG132 treatment. Finally, MG132‐mediated hyperexpression of ING5, PTEN, p53, Caspase‐3, Bax, and p27 suggested that the proteasomal pathway may degrade these proteins.

Similar to SAHA treatment, ING5 overexpression was confirmed to lower cell viability, energy metabolism, migration, and invasion and to promote the apoptosis of SH‐SY5Y cells, which is consistent with other reports.^41^, ^42^, ^43^, ^44^ Furthermore, the same regulatory effects of ING5 were observed on phenotype‐related protein expression (eg, acetyl‐histone upregulation). ING5 can form HAT complexes and subsequently promote histone acetylation.^8^ We performed Co‐IP, ChIP, and double‐ChIP assays and found that SAHA exposure and ING5 overexpression promoted the recruitment of ING5 and acetyl‐histones H3 and H4 to *p21*,* p27, CyclinD1*,* c‐myc,* and *Nanog* promoters by forming complexes through protein‐protein interactions. Therefore, we speculate that SAHA may upregulate ING5 expression in neuroblastoma cells to acetylate histones via HDAC inhibition or ING5 overexpression. Subsequently, ING5 can bind to these acetylated histones for transcriptional regulation in neuroblastoma cells.

According to previous research, miR‐1307, miR‐331‐3p, miR‐193a‐3p, and miR‐196a can promote ovarian cancer chemoresistance, hepatocellular carcinoma proliferation, and the DNA damage response and chemosensitivity of bladder cancer cells, and the anti‐apoptosis, invasion, and proliferation of pancreatic cancer cells via downregulated ING5 expression.^45^, ^46^, ^47^, ^48^ Wang et al^49^ found that miR‐193 promoted the proliferation of bone mesenchymal stem cells after low‐level laser irradiation treatment through ING5. In the present study, we found that SAHA may decrease miR‐640, miR‐543, miR‐624‐3p, and miR‐196‐b expression. However, only miR‐543 and miR‐196‐b overexpression decreased ING5 protein expression in SH‐SY5Y cells, which was ameliorated by SAHA exposure. These findings indicated that SAHA treatment indirectly facilitated ING5 translation by restraining miR‐543 and miR‐196‐b in SH‐SY5Y cells.

Our study demonstrated that SAHA or ING5 promoted the acetylation of histones H3 and H4 in neuroblastoma cells. Minardi et al^50^ reported that acetylated histone H3 expression was obviously lower in tumor tissues of renal cell carcinoma (RCC) than that in adjacent normal tissues. Acetylated histones H3 was also lower in Grades 3 and 4 pT1a RCC compared to that in Grades 1 and 2 pT1a RCC, indicating that histone acetylation is an early event in RCC and correlated with tumor aggressiveness. Nucleocytosolic translocation and downregulation of ING5 were positively associated with carcinogenesis and subsequent progression of gastric cancer, colorectal cancer, and head and neck squamous carcinoma.^51^, ^52^, ^53^ Here, the expression of acetylated histones H3 and ING5 was closely related to neuroblastoma tumor size, suggesting that their aberrant expression impacts the tumor growth of neuroblastomas.

In conclusion, we showed that SAHA and MG132 were synergistically cytotoxic to neuroblastoma cells by promoting apoptosis and inhibiting proliferation, migration, invasion, and energy metabolism through both in vitro and in vivo studies. In SH‐SY5Y cells, SAHA may downregulate the expression of miR‐196‐b and miR‐543, which target and suppress ING5 translation. SAHA strengthened the acetylation of histones H3 and H4 by both upregulating ING5 and inhibiting HDAC activity. Acetylated histones H3 and H4 and ING5 were recruited to the promoters of *Nanog, c‐myc, CyclinD1, p21,* and *p27* to form complexes for transcriptional regulation (Figure 8). Therefore, the expression of these acetylated histones and ING5 may be involved in neuroblastoma tumor growth. Accordingly, SAHA and/or MG132 can potentially be used as chemotherapeutic agents for neuroblastoma in clinical practice.

**Figure 8:** Outline of SAHA's antitumor effects in neuroblastoma cells. SAHA exposure suppressed the expression of miRNAs and subsequently enhanced ING5 expression, while HDAC activity was weakened, promoting the acetylation of histones H3 and H4. In the nucleus, ING5 and acetyl‐histones H3 (Ac‐H3) and H4 (Ac‐H4) form complexes and bind to the promoters of *p21*,* p27*,* CyclinD1*,* c‐myc,* and *Nanog* for transcriptional regulation. Note: red arrow indicates up‐ and downregulation

## ACKNOWLEDGEMENT

Neuroblastoma cell lines were kindly presented by Professor Carol J Thiele (National Institutes of health, National Cancer Institute, USA). Dr. Li B (Toronto Sickkids, Canada) and Dr. Rong YX (Oncology Clinical Research at Takeda Oncology, USA) kindly helped to revise the draft.

## CONFLICT OF INTEREST

None declared.
